The article "Effect Observation of Optimized Individualized Nursing Care Applied to ICU Patients with Severe Pneumonia" was published in 2022. Journal: Emerg Med Int.

# Effect Observation of Optimized Individualized Nursing Care Applied to ICU Patients with Severe Pneumonia

**DOI:** 10.1155/2022/6529558

**Published:** 2022-11-10

**Authors:** Xianpeng Wang, Yimei Qiu, Ting Xu, Yufeng Chen, Chunxiao Ying

**Affiliations:** Department of Intensive Care Medicine, Lishui City People's Hospital, Lishui, Zhejiang 323000, China

## Abstract

**Purpose:**

This study aims to observe the effect of optimized individualized nursing care applied to intensive care unit (ICU) patients with severe pneumonia (SP).

**Methods:**

440 patients with SP admitted to the ICU of our hospital from January 2019 to June 2020 were provided with routine nursing care (group A), and 550 patients with SP admitted from July 2020 to December 2021 were provided with optimized individualized nursing care (group B). The blood lactate index and acute physiology and chronic health evaluation (APACHE II) scores before and after care were compared between the two groups. The WBC count recovery time, mechanical ventilation time, antipyretic time, and length of hospital stay of the two groups were recorded. The complication rate of the two groups during the nursing care period was compared. The prognosis effect of the two groups after 6 and 12 months of discharge was followed up with the Seattle angina pectoris questionnaire (SAQ).

**Results:**

After care, the lactate level and lactate clearance rate were higher in both groups than before care, and the lactate level in group B was lower than that in group A and the lactate clearance rate was higher than that in group A (*P* < 0.05). After care, APACHE II scores were lower in both groups than before care, and lower in group B than in group A (*P* < 0.05). After care, the WBC count recovery time, mechanical ventilation time, antipyretic time, and length of hospital stay were shorter in group B than in group A (*P* < 0.05). During the nursing care period, the complication rate was lower in group B (5.82%) than in group A (11.59%) (*P* < 0.05). 6 and 12 months after discharge, the SAQ scores were higher in group B than in group A (*P* < 0.05).

**Conclusion:**

Optimized individualized nursing care applied to ICU SP patients can effectively improve the patients' physiological indicators, reduce complications, improve the prognosis of quality of life, and have a positive effect on the patients' speedy recovery.

## 1. Introduction

Severe pneumonia (SP) is a common acute and critical illness, mostly in the elderly. Patients are severely ill, progress rapidly, and have a poor prognosis, and some patients may even suffer from complications, such as infectious shock [1], acute respiratory distress syndrome [2], gastrointestinal bleeding [3], and multiorgan failure [4], leading to reduced survival rates. The main manifestations of the patient are edema and congestion in the lung tissue. In addition, the secretion in the respiratory tract is significantly increased compared with that before the disease, which make it easy to block part of the bronchioles and affects the gas exchange in the alveoli, thus hindering the patient's breathing [5]. The key to the treatment of this disease is to increase the effective oxygen intake, reduce the CO_2_ retained in the lungs, and keep breathing unobstructed. ICU monitoring is often used in the clinic to improve the treatment effect [6]. Martin-Loeches et al. [7] believe that scientific and reasonable nursing care measures can improve the clinical symptoms of patients from both physiological and psychological aspects and improve the quality of life. Individualized nursing care comprehensively implements the idea of serving patients, which emphasizes patient-centredness and expands the purely technical operation of nursing to include all aspects of patients' physiology, psychology, and spirituality, and provides patients with quality nursing services in a targeted manner. Especially in terms of health education for patients, nursing techniques and services, the number of nurses' rounds, and nurses' work attitudes, these measures have brought nursing close to patients and to the clinic, which has greatly brought the doctor-patient relationship closer, reduced medical disputes, and facilitated the recovery of patients' conditions. In this study, we adopted an optimized individualized nursing care intervention by evaluating the changes in blood lactate levels, acute physiology, and chronic health assessment system (APACHE II) scores, and Seattle angina survival quality scale (SAQ) scores in SP patients after the adoption of nursing care interventions to determine the impact of optimized individualized nursing care on the prognosis of SP patients, so as to accumulate experience for rational nursing care interventions in ICU SP patients.

The article "Effect Observation of Optimized Individualized Nursing Care Applied to ICU Patients with Severe Pneumonia" was published in 2022. Journal: Emerg Med Int.

## 2. Materials and Methods

### 2.1. Research Object

This study is a controlled historical experiment. The cases collected were 990 patients with SP admitted to our ICU between January 2019 and December 2021. Inclusion criteria: who all met the diagnostic criteria of the Chinese College of Emergency Physicians (CCEP) for SP [8] and were confirmed by clinicopathology; all patients were first cases, admitted to the hospital within 2 weeks of onset, and received reasonable treatment after admission; they were mentally and cognitively normal and able to cooperate effectively with treatment and rehabilitation care; patients or their families who had signed the relevant informed consent form. Exclusion criteria: persons with serious diseases of the cardiovascular system; persons suffering from malignant tumours; persons with severe immune system disorders; persons suffering from respiratory failure; persons suffering from coagulation disorders; those who had recently undergone major surgical treatment; persons with restricted mobility; those who died during nursing care and follow-up. 440 patients with SP admitted to the ICU of our hospital from January 2019 to June 2020 were provided with routine nursing care (group A), and 550 patients with SP admitted from July 2020 to December 2021 were provided with optimized individualized nursing care (group B). The general information collected from groups A and B was compared, and no statistical difference was found (*P* > 0.05), which is comparable (Table 1).

### 2.2. Care Methods

Patients in both groups received symptomatic support treatment, such as routine oxygenation, sputum evacuation, anti-infection, nutritional support, correction of water-electrolyte disturbances, acid-base balance, and active treatment of underlying diseases.

#### 2.2.1. Group A Was Provided with Routine Nursing Care

① Environmental care: nursing staff should keep the air in the ward clean with appropriate room temperature and humidity and regular ventilation. Also, ensure that the beds are neat and clean, the room is disinfected regularly, and the quietness of the ward is maintained. ② Daily care: healthcare workers should make detailed observations and records of changes in the patient's condition, advise the patient to take medication on time, arrange rest time reasonably, conduct daily vital sign checks for the patient, and perform regular oral, nasal, and suction care. ③ Health education: health care staff should develop relevant health education programmes in a targeted manner. For those with a high literacy level, they could communicate with patients by using the treatment means of the disease, the nursing programme, and precautions as entry points; for those with a low literacy level, the nursing staff should explain the knowledge of the disease in a simple and easy-to-understand manner to help patients establish a correct mindset towards the disease. ④ Discharge instruction: instruct patients to take appropriate physical exercise to improve their physical fitness and quality of life.

#### 2.2.2. Group B Was Provided with Optimized Individualized Nursing Care

① Enhance respiratory management: help the patient lie flat and pad the neck and back, and pay attention to clearing the oral and nasal secretions at any time to keep the respiratory tract unblocked. For those whose sputum was thick and difficult to cough up, Mucosolvan and normal saline were given for atomization inhalation to dilute the sputum. Sputum aspiration could be performed on anyone with SpO_2_ below 90%, elevated airway pressure and sputum sounds, and the patient's vital signs and parameters were closely monitored during aspiration. For older, weaker coughs and severe conditions, postural drainage might be used. For patients on ventilator-assisted ventilation, airway humidification should be enhanced to dilute sputum to prevent blockage of the tube. ② Oxygen therapy care: for patients with symptoms of hypoxia, blood oxygen saturation should be monitored, and an appropriate oxygen inhalation mode should be selected according to the results. Oxygen flow should be controlled at 5 L/min. For patients with CO_2_ retention, oxygen should be maintained at a low flow rate and be continuous, with an oxygen concentration of 30%–35% being appropriate. Also, during oxygen therapy care, the nurse must closely monitor the patient's respiratory rate and state of consciousness. ③ Bacterial culture and drug sensitivity test: bacterial cultures were regularly performed on airway secretions, and drug sensitivity tests were conducted on isolated pathogenic bacteria to keep track of changes in pathogenic bacteria and to select sensitive antibacterial drugs, pay attention to the duration of each use of antibacterial drugs within 8 d, and change the type of antibacterial drugs when appropriate to reduce bacterial resistance. ④ Complication prevention and control care: if patients develop cardiac insufficiency, they should be promptly treated with oxygen and sedation to control their condition. If there was no significant improvement in symptoms and the patient became agitated and cyanotic, appropriate resuscitation measures should be taken to prevent heart failure from developing. If patients develop symptoms of renal insufficiency, caregivers must closely monitor the patient's progress. ⑤ Psychological care and health education: SP patients often had symptoms, such as chest tightness and wheezing, and were accompanied by a sense of near-death, which, together with being in an ICU environment, further aggravated the patients' psychological burden and fear. Patients were provided with reasonable psychological guidance and health education, introduced to the purpose of various treatments and examinations and the methods of cooperation so that they could have a scientific understanding of their condition, reduce unnecessary psychological pressure, alleviate their anxiety and tension, and improve compliance with treatment.

The article "Effect Observation of Optimized Individualized Nursing Care Applied to ICU Patients with Severe Pneumonia" was published in 2022. Journal: Emerg Med Int.

### 2.3. Research Indicators

#### 2.3.1. Blood Lactate Indicator

Before and after care, a blood gas biochemistry analyser (Nova Stat Profile, USA) was used to measure lactate levels in both groups and to calculate the lactate clearance rate. Lactate clearance rate = (initial lactate level − post-treatment lactate level)/initial lactate level × 100%.

#### 2.3.2. APACHE II Score

Before and after care, APACHE II scores were tallied for both groups. It consists of 3 parts: the acute physical status score, age, and chronic health status score, with a total score of 71, 0–15 being nonserious, and >15 being serious, with lower scores indicating a less serious condition.

#### 2.3.3. Relevant Time Indicator

The WBC count recovery time, mechanical ventilation time, antipyretic time, and length of hospital stay of the two groups were recorded.

#### 2.3.4. Complication Rate

The occurrence of complications (such as infectious shock, pulmonary oedema, bronchiectasis, renal insufficiency, cardiac insufficiency, etc.) during care was recorded in both groups.

#### 2.3.5. Prognostic Effect

The prognosis effect of the two groups after 6 and 12 months of discharge was followed up with the SAQ. The assessment dimensions include activity limitation, disease onset, and quality of life, all of which are scored out of 100, with higher scores indicating better survival status.

### 2.4. Statistical Analysis

SPSS 22.0 was used for data analysis. The measurement data (±*s*) were tested by independent samples *t*-test. Count data *n* (%) was tested by *χ*^2^. A difference of *P* < 0.05 was considered statistically significant.

## 3. Result

### 3.1. Blood Lactate Indicator

After care, the lactate level and lactate clearance rate were higher in both groups than before care, and the lactate level in group B was lower than that in group A and the lactate clearance rate was higher than that in group A; the differences were statistically significant (*P* < 0.05). (Figure 1).

### 3.2. APACHE II Score

After care, APACHE II scores were lower in both groups than before care, and lower in group B than in group A; the differences were statistically significant (*P* < 0.05). (Figure 2).

### 3.3. Relevant Time Indicator

After care, the WBC count recovery time, mechanical ventilation time, antipyretic time, and length of hospital stay were shorter in group B than in group A; the differences were statistically significant (*P* < 0.05). (Figure 3).

### 3.4. Complication Rate

During the nursing care period, the complication rate was lower in group B (5.82%) than in group A (11.59%); the difference was statistically significant (*P* < 0.05). (Figure 4).

### 3.5. SAQ Score

Six and 12 months after discharge, activity limitation, disease onset, and quality of life scores in the SAQ were higher in group B than in group A; the differences were statistically significant (*P* < 0.05). (Figure 5).

The article "Effect Observation of Optimized Individualized Nursing Care Applied to ICU Patients with Severe Pneumonia" was published in 2022. Journal: Emerg Med Int.

## 4. Discussion

Pneumonia is an inflammation of lung tissue (fine bronchial, alveolar, and interstitial), caused by different etiologies and different pathogenic bacteria in different settings with similar or identical pathophysiological processes, all of which can deteriorate and worsen into SP when they develop into certain disease stages, causing multiorgan dysfunction or even being life-threatening, with a mortality rate of up to 30%–50% [9]. SP is prone to a variety of comorbidities and increases the financial burden of healthcare. In general, the treatment of this disease is the first choice of strong broad-spectrum antibiotics in sufficient amounts, and combined medication and ICU monitoring can significantly improve its efficacy [10]. In a way, appropriate nursing interventions are also of great therapeutic importance for the relief of the disease. Xin [11] showed an overall treatment effectiveness rate of 95.00% in elderly SP patients after anticipatory care intervention, which was significantly higher than that of the control group. Liu [12] showed significant improvement in blood gas analysis and family satisfaction after intensive care of a newborn with SP and respiratory failure. In this study, we adopted an optimized individualized nursing care plan, focusing on the implementation of targeted care according to the patient's specific condition, closely observing the changes in the patient's monitoring indicators during nursing care, and adjusting the nursing care plan according to the changes in the condition in a timely manner, which also achieved satisfactory results.

### 4.1. Optimized Individualized Nursing Care can Improve Physiological Indicators in ICU SP Patients

Patients with SP have congested and oedematous lung tissue, as well as increased respiratory secretions, which can lead to fine bronchial and bronchial obstruction, causing respiratory distress [13]. Lactate, a product of glucose anaerobic metabolism, reflects the degree of tissue hypoxia and intertissue perfusion levels and is a commonly used indicator to assess the severity of disease [14]. Tang et al. [15] concluded that individualized nursing interventions can improve pulmonary ventilation and reduce cellular hypoxia in patients with SP, thereby reducing abnormalities in pyruvate metabolism and resulting in lower lactate levels. Shadvar et al. [16] also concluded that for patients with SP in the ICU, care can be graded accordingly based on lactate clearance rate, thus shifting the original empirical judgement of the condition to an objective indicator, and that reasonable nursing interventions can improve blood lactate levels. In this outcome, after care, the lactate level and lactate clearance rate were higher in both groups than before care, and the lactate level in group B was lower than that in group A and the lactate clearance rate was higher than that in group A. It is suggested that optimized individualized nursing care can significantly improve hypoxic symptoms and intertissue perfusion in SP patients. This may be due to the fact that in optimized individualized nursing care, giving patients oral, nasal, and other respiratory care will effectively remove oral and nasal secretions and ensure the patency of the upper respiratory tract; giving patients symptomatic treatment such as sputum aspiration and oxygen inhalation can fully remove the obstruction of the lower respiratory tract, increase the oxygen saturation in the body, and improve the blood circulation; as a result, the patient's symptoms of dyspnoea improved, and the arterial blood lactate level decreased and lactate clearance increased. On the other hand, in group A, where only symptomatic treatment was administered, care was less effective than in group B because the nursing staff did not fully understand the changes in the patient's condition, resulting in inadequate care.

The article "Effect Observation of Optimized Individualized Nursing Care Applied to ICU Patients with Severe Pneumonia" was published in 2022. Journal: Emerg Med Int.

APACHE II score is an internationally used method to classify and assess the condition of critical patients and predict the prognosis, and it is also applicable to the assessment of the severity and prognosis of ICU patients [17]. Also, the higher the score, the more severe the patient's condition. After care in this study, APACHE II scores were lower in both groups than before care, and lower in group B than in group A. It is suggested that optimized individualized nursing care can speed up the recovery of ICU SP patients. This was also confirmed by the fact that the time to normalise the WBC count, the time for mechanical ventilation, the time for fever reduction, and the length of stay in the hospital were shorter in group B than in group A after care in this study. Analyze the reasons for the above results, which may be related to the following points: First, in the process of strengthening respiratory management and oxygen therapy care, individualized care measures were developed according to the patient's condition, a comprehensive understanding of the patient's needs was gained and symptomatic care was given so that the patient's condition was effectively controlled and the risk to life was reduced. Second, in the past, the clinical application of antibiotics was mostly empirical, which not only had a poor therapeutic effect but also easily led to bacterial resistance. This study strengthens the identification of pathogenic bacteria and the timely use of narrow-spectrum antibiotics after identifying the pathogenic bacteria, so as to prevent dysbiosis and fungal infection caused by the enhancement of bacterial resistance due to the long-term use of broad-spectrum antibiotics, which plays an important role in controlling the progress of patients' diseases and shortening the recovery time. Third, through health education, patients can also learn what to look out for in their daily lives and reduce fluctuations in their condition caused by their own factors and poor lifestyle habits. Finally, through comprehensive disease promotion and psychological care, patients have a detailed understanding of their condition and the treatment process, which can alleviate the psychological barriers that exist in their treatment, thus improving treatment compliance and facilitating recovery.

The article "Effect Observation of Optimized Individualized Nursing Care Applied to ICU Patients with Severe Pneumonia" was published in 2022. Journal: Emerg Med Int.

### 4.2. Optimized Individualized Nursing Care can Reduce Complications and Improve Prognostic Life Quality in ICU SP Patients

ICU SP is mostly seen in elderly patients, whose immune systems are low and whose organ reserve function is relatively poor. Once the disease progresses, it can lead to rapid failure of all organ functions that are barely in equilibrium in a short period of time, and can easily lead to various complications and seriously affect the patient's prognosis [18, 19]. Based on this, it is of great significance to strengthen the prevention and treatment of complications in the nursing process for SP patients in the ICU. During the nursing period of this group, the complication rate of group B was 5.82%, significantly lower than that of group A at 11.59%. It is suggested that optimizing individualized nursing is an effective nursing method to reduce the related complications of SP patients during ICU treatment, which is basically consistent with the research conclusion of Chen [20].

SAQ is a recognized, effective index to evaluate the results of clinical treatment measures and has been widely used in the evaluation of the quality of life of patients with coronary heart disease [21]. In this study, it was applied to the long-term prognosis evaluation of discharged patients with severe pneumonia. The results showed that 6 and 12 months after discharge, the SAQ scores in group B were higher than those in group A. This may be due to the fact that health education in optimized individualized nursing care compensates for the lack of health education for patients after discharge, significantly improves the patient's activity limitation and disease onset, and improves the patient's quality of life. This proactive model of care not only fosters a sense of achievement and self-discipline among caregivers but also improves the patient's postdischarge status and can maximise the patient's prognosis for a better quality of life.

The article "Effect Observation of Optimized Individualized Nursing Care Applied to ICU Patients with Severe Pneumonia" was published in 2022. Journal: Emerg Med Int.

In summary, the optimized individualized nursing care applied to ICU SP patients can effectively improve the patients' physiological indicators, reduce complications, improve the prognosis of quality of life, and have a positive effect on the patients' speedy recovery.

## Figures and Tables

**Figure 1:** Blood lactate indicator. *Note*. (a). Lactate level (mmol/L). (b). Lactate clearance rate (%). ^*∗*^and ^△^represent a comparison with the same group before care and group A after care, respectively, *P* < 0.05.

**Figure 2:** APACHE II score. *Note*. ^*∗*^and ^△^represent a comparison with the same group before care and group A after care, respectively, *P* < 0.05.

**Figure 3:** Relevant time indicators. *Note*. (a). WBC recovery time. (b). Mechanical ventilation time. (c). Antipyretic time. (d). Length of hospital stay. Comparison with group A, ^△^*P* < 0.05.

**Figure 4:** Incidence of various complications. *Note*. Comparison with group A ^△^*P* < 0.05.

**Figure 5:** SAQ score. *Note*. (a). Activity limitation (scores). (b). Disease onset (scores). (c). Quality of life (scores). Comparison with group A, ^△^*P* < 0.05.

**Table 1:** General information for groups A and B.

Items	Group A (*n* = 440)	Group B (*n* = 550)	*χ* ^2^/*t*	*P*
Age (years old)	66.86 ± 7.43	66.01 ± 7.37	1.797	0.073

Disease duration (*d*)	11.95 ± 7.04	11.71 ± 5.64	0.596	0.552

Gender (*n*, %)				
Male	258 (58.64)	294 (53.45)	2.661	0.103
Female	182 (41.36)	256 (46.55)		

Basic diseases (*n*, %)				
Hypertension	165 (37.50)	210 (38.18)	0.048	0.826
Diabetes	86 (19.55)	120 (21.82)	0.766	0.381
Coronary heart disease	80 (18.18)	122 (22.18)	2.408	0.121
Chronic obstructive pulmonary disease	72 (16.36)	86 (15.64)	0.096	0.756
Cerebral infarction	50 (11.36)	60 (10.91)	0.051	0.821
Cerebral haemorrhage	42 (9.55)	49 (8.91)	0.119	0.731
Others	205 (46.59)	242 (44.00)	0.663	0.416

## Data Availability

The data used in the current study are available from the corresponding author.
